The article "Study on the Relationship between Lung Cancer Stromal Cells and Air Cavity Diffusion Based on an Image Acquisition System" was published in 2022. Journal: Contrast Media Mol Imaging.

# Study on the Relationship between Lung Cancer Stromal Cells and Air Cavity Diffusion Based on an Image Acquisition System

**DOI:** 10.1155/2022/2492124

**Published:** 2022-07-14

**Authors:** Shan Bai, Zhi Wang, ZhiHong Sun, Zhuo Liu

**Affiliations:** ^1^Department of Thoracic Surgery, The Hospital of Xidian Group, No. 97 FengDeng Rd, Xian, Shaanxi 710077, China; ^2^Department of Emergency, The Second Affiliated Hospital of Xi'an Medical University, 167 Fangdong Road, Xian, Shaanxi 710038, China; ^3^Department of Thoracic Surgery, The Second Affiliated Hospital of Xian Medical University, 167 Fangdong Road, Xian, Shaanxi 710038, China; ^4^Department of Emergency, The Hospital of Xidian Group, No. 97 FengDeng Rd, Xian, China

## Abstract

**Objective:**

The study aimed to investigate the role of tumor stromal cells in the pathogenesis of STAS, the relationship between air diffusion (STAS) and tumor stromal cells (TSCs) was studied, and the prognostic significance of TSC and STAS in patients with lung adenocarcinoma was evaluated.

**Methods:**

A total of 150 patients with lung cancer diagnosed in the Affiliated Hospital of Jiangsu Province were selected. From the perspective of pathology, medical information technology was used to assist the diagnosis. The data of multiple magnetic resonance images were analyzed by three-dimensional space convolution (CNN), fuzzy neural network (FNN), transfinite learning machine (ELM), and binarization.

**Result:**

After data fusion, the specificity and sensitivity of multiple magnetic resonance (MRI) data are significantly higher than those of single MRI data, and the more fusion times, the better the sensitivity and specificity. With the increase in the number of information and data fusion, the proportion of the significant effect and the comprehensive effective rate of patients are on the rise. Multiple MRI data fusion examination and analysis under medical information technology can improve the cure rate of patients, and the 1-year survival rate and the 3-year survival rate of patients have also gradually improved.

**Conclusion:**

The MRI data fusion diagnosis method under the application of information technology can improve the sensitivity and specificity of the diagnosis results and comprehensively improve the clinical cure rate and the survival rate at different times of prognosis. In the context of the current big data information age, this multifeature fusion analysis technology is playing a more and more important role in medical treatment. The application of this method and technology not only improves the quality of life of patients but also processes multiple types of data at one time only by using the proposed medical assistant diagnosis model, which can save the diagnosis time to a certain extent. It has effectively realized the medical management and medical service quality and has important promotion significance.

The article "Study on the Relationship between Lung Cancer Stromal Cells and Air Cavity Diffusion Based on an Image Acquisition System" was published in 2022. Journal: Contrast Media Mol Imaging.

## 1. Introduction

With the continuous development of medical technology, the screening rate and the cure rate of early cancer are also increasing, but lung cancer accounts for a large proportion of cancer deaths. In the global cancer data statistics in 2020, about 1.8 million people died of lung cancer [1]. The main cause of death of lung cancer is non-small-cell lung cancer (NSCLC). Its incidence rate and mortality rate are relatively high. Lung adenocarcinoma is a common form of NSCLC, and its incidence rate is about half of what mentioned in [2]. Previous researchers mainly focused on the malignant cells of cancer. With the in-depth study of lung adenocarcinoma and the study of pathological features such as molecular biology, immunohistochemistry, and morphological characteristics of cancer, researchers found some new morphological features to predict the prognosis and treatment of patients. Air cavity diffusion (STAS) refers to that a single cell of a tumor enters the lung parenchyma from the edge of the tumor through the air cavity. As a new way of metastasis of lung cancer, it can predict the recurrence and survival of lung adenocarcinoma [3]. STAS is the diffusion of lung cancer cells in the lung parenchyma beyond the edge of the main tumor. However, STAS is not only a prognostic factor independent of the growth pattern but also an independent risk factor for local and distant recurrence after local resection of stage I lung adenocarcinoma. Therefore, judging the existence of STAS before or during operation is of a great-guiding significance for the selection of surgical methods and postoperative treatment of lung adenocarcinoma. At present, the research on STAS has become a hot topic. The existence of STAS is not only related to lung cancer histopathology, gene mutation, and other factors but also confirmed by many studies that it can be used as an independent factor related to tumor recurrence and prognosis [1]. Previous studies have shown that the tumor microenvironment has an important impact on the survival of cancer cells. The tumor microenvironment includes tumor cells themselves and a variety of stromal cells, including various inflammatory cells, as well as newly formed microvessels due to tumors [4]. These stromal cells have important effects on the reproduction, survival, and invasion of tumor cells.

The development of intelligent computing technology has driven the application of an intelligent auxiliary system in all walks of life, and a large number of clinical symptoms, image examination, and other data are required in the diagnosis process of students in traditional Chinese medicine hospitals. Using medical information technology to assist diagnosis can use more comprehensive information to improve the accuracy of diagnosis and reduce the error of diagnosis [5].

The article "Study on the Relationship between Lung Cancer Stromal Cells and Air Cavity Diffusion Based on an Image Acquisition System" was published in 2022. Journal: Contrast Media Mol Imaging.

At present, there is no relevant report on the mechanism of tumor air diffusion (STAS). The purpose of this study is to study and explore how to use medical information technology to study the relationship between STAS and tumor stromal cells (TSC) from the perspective of pathology and to explore the role of tumor stromal cells in the pathogenesis of STAS. In traditional diagnostic methods, doctors' diagnosis is entirely a subjective judgment process, which will be limited and affected by the experience and knowledge level of diagnostic doctors. Moreover, doctors are prone to omit some details when making diagnosis. The objective judgment of computers has great advantages in correcting these errors and deficiencies.

## 2. Journals Reviewed

Chen Donglai et al. studied the air cavity diffusion of lung cancer. In 2015, the World Health Organization introduced the concept of air cavity invasion. STAS is an important part of it. It is the diffusion of lung cancer cells from the lung parenchyma to outside the main boundary of the tumor through airway diffusion. It often occurs in lung cancer, especially early lung adenocarcinoma [6]. STAS is a newly discovered invasive mode of lung adenocarcinoma, and STAS is closely related to the recurrence and survival of lung cancer, but it is very difficult to predict and evaluate STAS [7]. Yoshida et al. analyzed 709 patients with lung adenocarcinoma, performed immunohistochemical analysis, and used the chi-square test to analyze variables to explore the relationship between immune cell infiltration and STAS. The results showed that in resected lung adenocarcinoma, the infiltration of relevant macrophages in the tumor immune microenvironment was related to the higher speed of tumor passing through STAS [8]. In NSCLC, cancer cells spread through STAS, which has a negative impact on the prognosis of patients, but the preoperative diagnosis of STAS is very difficult. Onozato Yuki et al. used radiomics combined with machine learning to establish a model and tried to predict and analyze STAS [9]. Qi et al. extracted texture features from 216 patients with lung adenocarcinoma by using morphological analysis and radiation features around and in the nodules of chest CT images, established radiation models and compared them, and compared the diagnostic efficiency of STAS in lung adenocarcinoma [10]. Okan et al. selected 63 patients with lung adenocarcinoma undergoing pneumonectomy, calculated the parameters, evaluated the STAS of pathological samples, and discussed the prediction of STAS in patients with lung adenocarcinoma by preoperative 18F-FDG PET/CT imaging so as to achieve the role of adjuvant therapy [11]. Liu and Wang carried out high-resolution CT examination for patients with different lesions, analyzed its impact characteristics and clinical value, and summarized and analyzed the differences in high-resolution CT impact characteristics of simultaneous multiple primary lung adenocarcinoma and intrapulmonary metastasis in lung adenocarcinoma classes [12]. The diagnostic accuracy of the single-phase imaging system is poor because of the poor relationship between the diagnostic accuracy of the single-phase imaging system and the actual diagnosis of lung cancer.

The article "Study on the Relationship between Lung Cancer Stromal Cells and Air Cavity Diffusion Based on an Image Acquisition System" was published in 2022. Journal: Contrast Media Mol Imaging.

With the development of intelligent technology, information technology is being gradually applied to medical institutions. Based on the application of this technology, the hospital can establish a more complete set of the medical data storage system [13]. Using its medical data fusion analysis technology for analysis and then using the auxiliary evaluation of imaging system equipment to evaluate the results of diagnosis and treatment can increase the diagnostic accuracy.

## 3. Medical Information Technology-Assisted Diagnosis of TSC and STAS in Lung Cancer

Imaging recognition technology plays a key role in the analysis and diagnosis of the relationship between TSC and STAS in lung cancer. At present, the best application effect is the application of magnetic resonance imaging technology. Magnetic resonance imaging is a kind of research on tomography. Through the principle of magnetic resonance, it can use the phenomenon of magnetic resonance to obtain the electromagnetic signal of the corresponding part of the human body from the human body, reconstruct the human body feature information according to the signal, and conduct research and analysis of different data by fusing multimodal image features.

Relevant network information data features such as human cortical thickness, bone density, consistency and dissimilarity of parts can be extracted from the structural image and the static function image of magnetic resonance. The detailed magnetic resonance image information data can be obtained by detecting the electromagnetic wave emitted by the external magnetic field. The data fusion analysis of multiple MRI images is shown in Figure 1:

In Figure 1, the logical framework of the data fusion analysis algorithm for patients with multiple examinations of magnetic resonance images is shown. Multiple magnetic resonance (MRI) imaging three-dimensional vector models, respectively, collect the corresponding imaging data information for multiple three-dimensional vector models and then expand the three-dimensional space convolution (CNN) to strengthen the data edge. After obtaining the enhanced data, fuzzy neural network (FNN) and transfinite learning machine analysis (ELM) are performed, respectively, After CNN, FNN, and ELM are performed for all image information, the second round of centralized FNN analysis is carried out. After binarization (BIN), the output information result is output of the evaluation result of air cavity diffusion of a lung cancer stromal cell tumor. The closer the data result is to 1.000, the greater the probability of air cavity diffusion is considered.

The article "Study on the Relationship between Lung Cancer Stromal Cells and Air Cavity Diffusion Based on an Image Acquisition System" was published in 2022. Journal: Contrast Media Mol Imaging.

## 4. Data and Methods of Clinical Trials

### 4.1. General Information of Patients

A total of 150 patients with lung cancer diagnosed in the Affiliated Hospital of Jiangsu from March 2020 to March 2021 were selected, including 86 males and 64 females, with an average age of 34∼68 years. The number of smokers accounted for 60.7%.

Inclusion criteria were as follows: patients with lung tumors diagnosed by the hospital, and the relevant data and physical conditions should meet the standards of admission.

Exclusion criteria were as follows: patients with multiple complications, patients receiving neoadjuvant radiotherapy and chemotherapy, and patients with incomplete data and information.

### 4.2. Traditional MRI Diagnostic Methods

All 150 patients need to perform the enhanced MRI examination of the lungs on schedule. The single result after the examination is recorded in the medical information big data system with the imaging three-dimensional vector model, and then, the diagnosis and treatment results are evaluated with the assistance of the MRI-assisted diagnosis expert system (provided by the MRI equipment).

### 4.3. MRI Data Fusion Diagnosis Method

All 150 patients need MRI examination on schedule many times. The imaging results after multiple examinations are analyzed by using the MRI data fusion analysis technology designed in this study, and the expert system provided is used to assist multiple fusions to evaluate the diagnosis and treatment results.

### 4.4. Observation Contents and Statistical Methods

We analyze the single MRI data results of the patients used, analyze the information data results of multiple MRI examinations and imaging fusion of the patients used, and observe the comparative analysis of multiple MRI results after multiple superposition fusions, and single MRI data results, as well as the impact on lung cancer tumor stromal cells and air cavity diffusion.

The article "Study on the Relationship between Lung Cancer Stromal Cells and Air Cavity Diffusion Based on an Image Acquisition System" was published in 2022. Journal: Contrast Media Mol Imaging.

The above medical information technology needs to use a variety of neural network basis function calculation formulas in the application of MRI, among which, the spatial convolution basis function of MRI image data processing is analyzed, as shown in formula (1):

(1) $$\begin{array}{c} y=\int_{-\infty }^{+\infty }g\left(x\right)j\left(a-x\right)\text{d}x. \end{array}$$

Where*g*(*x*) is the original image of the collected data, *j*(*a* − *x*) is the convolution kernel of the basis function, *a* is the positioning variable, and *y* is the output value of the neural network;

If FNN is used to control the recent change law of time series data, it is necessary to analyze the basis function of the sixth-order polynomial depth iterative regression FNN algorithm based on the FNN to enrich the change law of the complex function curve, as shown in formula(2):

(2) $$\begin{array}{c} y=\sum_{i=1}^{n}\sum_{j=0}^{5}A_{j}x_{i}^{j}. \end{array}$$

Where *A*_*j*_ is the coefficient to be regressed of the *j* th order iterative function polynomial and *j* is the order of the iterative function polynomial;

The statistical significance of the ELM application is to analyze the changes in periodic data. The ELM calculation formula is as follows(3):

(3) $$\begin{array}{c} y=\sum_{i=1}^{n}\left[A\cdot \;\sin\left(Bx_{i}+C\right)+D\right]. \end{array}$$

Where *i* is the value of the pointer variable, *n* is the node function of the upper neural network, and A. B, C, and D are the regression variables of the basis function.

The bin neural network basis function formula is as follows(4):

(4) $$\begin{array}{c} y=\sum_{i=1}^{n}\frac{1}{A+B\cdot e^{x_{i}}}. \end{array}$$

Where *e* is the natural basis function constant and the meanings of other symbols are the same as previously mentioned.

## 5. Clinical Trial Results and Discussion

### 5.1. Diagnostic Sensitivity and Specificity of STAS in Pulmonary Interstitial Cell Carcinoma

Interstitial cell carcinoma is an important cancer in lung cancer. Its biological characteristics and particularity are determined by the substantive factors causing cancer. The interstitial components of cancer are not specific and mainly play a role in supporting and nourishing the essence of cell carcinoma. It is generally composed of connective tissue, blood vessels, and lymphatic vessels. Lung stromal cell cancer is also a tumor that changes the alveolar septum. A stromal tumor generally refers to a mesenchymal tumor on the gastrointestinal wall. The origin of this cell tumor is not easy to be clear, and its location is mostly located between organs. Its early clinical manifestations are not typical, which are often accompanied by abdominal pain and compression. STAS refers to micropapillary cell clusters, solid cell nests, or single tumor cells in the air cavity outside the boundary of the main tumor body In addition to the traditional concept of invasion of the pleura and interstitium (STAS), the fourth mode of invasion of pulmonary adenocarcinoma is determined as the invasion of the pleura. In order to study the difference in MRI three-dimensional imaging vector data information of the aforementioned patients, the diagnosis of pulmonary interstitial cell carcinoma STAS in different patients is analyzed and discussed. The comparison of diagnostic sensitivity and specificity of pulmonary interstitial cell carcinoma STAS is shown in Table 1.

The article "Study on the Relationship between Lung Cancer Stromal Cells and Air Cavity Diffusion Based on an Image Acquisition System" was published in 2022. Journal: Contrast Media Mol Imaging.

Table 1 shows the sensitivity and specificity comparison data of traditional MRI diagnostic methods and five MRI data fusion diagnostic methods. Through analysis and comparison, it can be seen that the sensitivity and specificity of MRI data fusion diagnostic methods are more accurate than those of traditional MRI diagnostic methods. It is obvious that the more fusion times, the more accurate the sensitivity and specificity data.

In order to intuitively analyze the sensitivity and specificity comparison results of two different MRI diagnostic modes, Table 1 is visualized and Figure 2 is obtained.

Table 1 and Figure 2 show the sensitivity and specificity data between the traditional MRI diagnosis method and MRI data fusion, 2 and MRI data, 3, 4, and 5 separate MRI data, and the more sensitivity and specificity results.

### 5.2. Clinical Cure Rates Based on the Two Diagnostic Modalities

MRI has obviously an imaging effect on nonbony parts or soft tissues of the human body and is less destructive to the human body. The application of MRI technology can more clearly see the spinal cord, the nerve, and the characteristics of different parts such as TSC, muscle, and other detected parts. When multiple image tests are needed for analysis and diagnosis, MRI is the best imaging method. It can use medical information technology to fuse and analyze data at different times to assist diagnosis and treatment. The image information observed by MRI assisted technology will be clearer and more comprehensive, and the quality of information results will also directly affect the quality of patients' visits. Observe the influence of two different diagnostic modes on the clinical efficacy of patients, as shown in Table 2:

In Table 2, we compare the prognostic effect of patient MRI alone and the multiple prognostic effects of MRI data fusion under medical information technology. Among them, the proportion of one MRI apparent effect under the fusion of medical information technology and the data of comprehensive response efficiency are not obvious compared with that of MRI alone. The t-value is <9.876. The *P* value is <0.03. The proportion of three MRI apparent effects under medical information technology fusion increased by 3.1% compared with MRI alone. Combined response efficiency is 2.9% higher than the data of MRI alone. Its t-value is <8.425. A *P* value is <0.01. There is already a clear gap between the two comparisons. The proportion of 5 MRI apparent effects under medical information technology fusion increased by 8.6% compared with MRI alone. Combined response efficiency improved by 7.6% over the data for MRI alone. And the t-value is <5.613. A *P* value is <0.008. There is already a significant gap between the two comparisons. The results show that with the superposition of information and data fusion time under medical information technology, the gap between the results of its information data and the results of a single MRI information data is also growing, with an extremely obvious statistical point of view.

The article "Study on the Relationship between Lung Cancer Stromal Cells and Air Cavity Diffusion Based on an Image Acquisition System" was published in 2022. Journal: Contrast Media Mol Imaging.

Clinical cure analysis results of TSC and STAS symptoms of lung cancer in different patients are shown in Figure 3.

Figure 3, shows that obviously, with the increase of the number of information data fusion, the curative effect and comprehensive efficiency of patients are gradually increasing. The research results show that the application of multi-MRI data fusion examination and analysis under medical information technology can significantly improve the curative rate of patients.

### 5.3. Prognostic Effect Based on Both Diagnostic Modalities

The detection analysis of MRI alone and the result analysis of the fusion amount of MRI detection data not only directly affect the clinical cure effect of patients but also affect the survival effect of patients at different times after cure. The survival rate analysis of patients observed at different times of prognosis in this study is summarized in Table 3.

The comparison of the prognostic survival effect at different times in the above two different diagnostic modes is shown in Figure 4.

Table 3 and Figure 4 show the analysis and comparison of MRI patient survival information data and data fusion, the one-year survival rate, and the 3-year survival rate compared with the MRI survival rate alone and the 3-year survival rate, and with the increase in data fusion times under medical information technology, the 1-year survival rate and the 3-year survival rate have gradually increased.

## 6. Conclusion and Future Direction

With the continuous reform of the medical system, medical information management has become the mainstream development trend. During the actual management work, major medical institutions apply computer information technology to form a perfect computer management system on the basis of meeting the information needs of various businesses, which can not only improve the efficiency of hospital medical information management but can also enable computer information technology to give full play to its functions. It is an important measure to promote the transformation of China's medical undertakings to the direction of informatization. The application of medical information technology can enable different patients to establish a systematic information data storage system based on clinical data, which can more intuitively present the complete medical data of patients. This study is mainly aimed at the correlation analysis of TSC and STAS for the diagnosis of lung cancer with the help of medical information technology. Through the logical framework of the data fusion analysis algorithm of magnetic resonance images after multiple tests, the research objects using traditional MRI diagnosis methods and MRI data fusion diagnosis methods are observed and analyzed in different aspects. The results showed that the MRI data fusion diagnosis method under the application of information technology could improve the sensitivity and specificity of the diagnosis results and comprehensively improve the clinical cure rate and the survival rate at different times of prognosis. The application of this method and technology not only improves the quality of life of patients but also realizes the medical management and medical service quality efficiently, which is of great significance for promotion.

The article "Study on the Relationship between Lung Cancer Stromal Cells and Air Cavity Diffusion Based on an Image Acquisition System" was published in 2022. Journal: Contrast Media Mol Imaging.

## Figures and Tables

**Figure 1:** Logical architecture of the data fusion analysis algorithm based on multiple magnetic resonance images.

**Figure 2:** Visualization plots comparing sensitivity and specificity of the two MRI diagnostic modalities.

**Figure 3:** Visual visualization of clinical cure rates for two different diagnostic modalities.

**Figure 4:** Comparison and visualization of the prognostic survival effects for the two different diagnostic modalities.

**Table 1:** **C**omparison of sensitivity and specificity of the two MRI diagnostic modalities.

Grouping		Sensitivity	Specificity
Alone MRI		95.2	83.7
Data fusion	1	95.8	84.1
	2	96.3	85.6
	3	96.9	88.7
	4	97.3	90.4
	5	97.9	93.3

**Table 2:** Comparison of the clinical cure rates for the two different diagnostic modalities.

Grouping		The proportion of effective	Comprehensive and efficient
Alone MRI		83.1	84.6
Data fusion	1	83.8	84.9
	2	84.5	85.1
	3	86.2	87.5
	4	89.5	90.3
	5	91.7	92.2

The article "Study on the Relationship between Lung Cancer Stromal Cells and Air Cavity Diffusion Based on an Image Acquisition System" was published in 2022. Journal: Contrast Media Mol Imaging.

**Table 3:** Comparison of prognostic survival outcomes between the two different diagnostic modalities.

Grouping		1-year survival rate	3-year survival rate
Alone MRI		69.4	70.1
Data fusion	1	72.3	72.8
	2	74.3	75.5
	3	78.5	80.4
	4	82.4	84.3
	5	86.3	89.7

## Data Availability

The data underlying the results presented in the study are available within the manuscript.
